The article "A rare case of Balo's disease in a young adult: A clinical presentation and management" was retracted in 2026. Reasons: fabricated or falsified data; plagiarized images; overlap with other authors' work; missing or withdrawn patient consent.

# A rare case of Balo's disease in a young adult: A clinical presentation and management

**DOI:** 10.1002/ccr3.8520

**Published:** 2024-02-09

**Authors:** Mansi Singh, Abeer Almusleh, Geethika Mandru, Snigdh Sahu, Ogbonnaya Akuma, Chinaza Mercy Akuma, Brinda Desai, Archit Kumar Nigam, F. N. U. Sandhiya, Manjeet Singh, Aadil Mahmood Khan

**Affiliations:** ^1^ Bogomolets National Medical University Kyiv Ukraine; ^2^ Alnajah National University Nablus Palestine; ^3^ Davao Medical School Foundation Davao City Philippines; ^4^ Ebonyi State University Abakaliki Nigeria; ^5^ Nnamdi Azikiwe University Awka Nigeria; ^6^ GMERS Medical College Valsad India; ^7^ Department of Radiodiagnosis Regency Hospital Kanpur Kanpur India; ^8^ Chandka Medical College Larkana Pakistan; ^9^ Clinical Research Fellow OSF St Francis Medical Centre Peoria Illinois USA

**Keywords:** Balo concentric sclerosis (BCS), Balo's disease, demyelinating disorders, magnetic resonance imaging (MRI), multiple sclerosis (MS)

## Abstract

**Key Clinical Message:**

Accurate diagnosis of rare neurological conditions like Balo's concentric sclerosis (BCS) is challenging but crucial for tailored treatment. Interdisciplinary collaboration and further research are essential to advance our understanding.

**Abstract:**

This case report presents a 32‐year‐old female patient with a puzzling neurological condition characterized by feverish feelings, joint pain, unclear speech, and an unsteady gait. Initial management did not lead to improvement, and further examination revealed neurological involvement and joint tenderness without signs of inflammatory arthritis. Laboratory investigations ruled out infectious and autoimmune causes. Magnetic resonance imaging (MRI) showed well‐defined lesions with concentric rings, leading to a diagnosis of Balo' concentric sclerosis. Treatment with intravenous methylprednisolone resulted in limited improvement. This case highlights the importance of thorough evaluation and collaboration in diagnosing rare neurological conditions. Further research is needed to enhance the understanding and treatment of rare neurological disorders.

## 1 INTRODUCTION

Baló's concentric sclerosis (BCS), also called Balo's disease, is a rare variant of multiple sclerosis (MS) characterized by severe monophasic demyelination.^1^ It is most seen in people with Filipino and Han Chinese ethnicity and less common in the Caucasian population.^2^ In the United States, MS affects 400,000 people.^3^ Due to the rarity, challenging variation in presentations, and availability of technology to achieve the diagnosis of BCS, accurate incidence rates have not been accurately documented. BCS occurrence is higher in males than females, with a wide range of presenting ages from 4 to 56 years old, with an average age of 36 years old.^4^, ^5^ Patients with BCS usually present with cognitive dysfunction, headache, paralysis, and muscle spasm.^6^

The symptoms of BCS and MS are almost similar except, that MS presents with more of a waxing and waning pattern while BCS tends to progress rapidly. The cause of BCS remains unknown. However, several studies suggest that it has an autoimmune etiology.^7^

The distinctive pathological features of this disease include extensive demyelinated lesions that display a unique arrangement characterized by alternating layers where myelin remains intact and others where it is damaged. This pattern may be attributed to a potential scenario where mild tissue injury occurs at the periphery of the expanding lesion. This injury could trigger the production of neuroprotective proteins, consequently, leading to the formation of alternating layers of myelin.^8^

These alternating myelin bands are identified on T2‐weighted images (T2WI) which show varying signal intensities of hyperintense lesion representing areas of demyelination and hypo/isointense representing normal myelinated white matter. The pattern will resemble a “whirlpool” with concentric rings, akin to the appearance of a “tree trunk” or “onion bulb”.^9^, ^10^ These bands disappear over time eventually. We present a case of A 32‐year‐old woman with a complex neurological condition, BCS, experienced fever, joint pain, speech issues, and unsteady gait. Despite initial treatment, methylprednisolone treatment provided limited improvement. BCS presents diagnostic challenges, emphasizing the need for accurate diagnosis and further research.

## 2 CASE PRESENTATION

This case report describes a 32‐year‐old female patient who presented with a puzzling neurological condition. The patient initially experienced feverish feelings and joint pain, which were followed by a sudden onset of unclear speech and unsteady gait. The initial management by a physician did not lead to improvement, prompting a referral.

On physical examination, the patient appeared fatigued and had a low‐grade fever. Her vital signs were as follows: temperature of 99.5 F (37.5°C), heart rate of 90 beats per minute, blood pressure of 120/80 mmHg, and respiratory rate of 16 breaths per minute.

A neurological examination revealed an unsteady gait with mild ataxia. The patient had difficulty maintaining balance while walking, exhibiting a wide‐based stance and slight swaying. She demonstrated dysarthria, with slurred and unclear speech. There were no signs of focal weakness or sensory deficits. Deep tendon reflexes were symmetric and normal. A joint examination revealed mild tenderness on palpation in both knees, with no signs of swelling or redness. The range of motion of all joints was within normal limits, and there were no signs of joint effusion or synovitis. The rest of the physical examination, including cardiovascular, respiratory, abdominal, and skin examination, was unremarkable. There were no signs of rash, lymphadenopathy, or hepatosplenomegaly.

These findings on physical examination were consistent with a central nervous system involvement, given the neurological symptoms and signs observed. The joint tenderness without obvious signs of inflammatory arthritis raised the possibility of an associated autoimmune component. On series of MRI images clearly demonstrates the presence of lesions in the left frontal lobe. On the T2‐weighted/STIR image (Figure 1A,B), the lesions are hyperintense, indicating increased water content. Additionally, on the diffusion‐weighted image (Figure 1C), the lesions show vivid diffusion restriction, indicating restricted movement of water molecules. The T1‐weighted image (Figure 1D) further reveals multiple well‐defined lesions in the left frontal lobe, with the largest lesion measuring 21 × 20 mm and exhibiting concentric rings. These lesions appear hypointense on T1 images. Overall, these images provide valuable insight into the nature and characteristics of the lesions in the left frontal lobe.

**FIGURE 1:** Left Frontal Lobe Lesions on MRI, (A and B) Hyperintense on T2‐weighted/STIR images, (C) Diffusion weighted (DW) observed, (D) Multiple hypointense lesions on T1‐weighted image.

Based on the perplexing neurological presentation, negative laboratory investigations, and characteristic MRI findings, a diagnosis of Balo's concentric sclerosis was made. The patient was started on intravenous methyl‐prednisolone therapy to reduce inflammation and mitigate disease progression. Although there was limited improvement in motor function and speech following treatment, the patient's condition stabilized, and further rehabilitation was planned to optimize her functional abilities.

## 3 DISCUSSION

BCS is an uncommon condition that was once assumed to be a fatal or poorly treated fulminant demyelinating disorder. However, there is a range of potential appearances for BCS lesions, including benign illnesses. BCS lesions may develop in people who already have MS or may signal the beginning of a demyelinating illness that may eventually resemble normal MS clinically and radiologically. When immunopathologic phenotyping was carried out, all lesions showed the oligodendrocytopathy pattern (Pattern III). Tissue ischemia and tissue preconditioning may cause BCS lesions to seem laminated; however, the mechanisms causing the distinctive concentric stacking are not well understood.^11^ Lesions that looked like Baló lesions had either a lamellar or mosaic pattern with patches of demyelinated and myelinated areas surrounding a larger demyelinated area, called the storm center, or a pattern of parallel rings with and without myelin. The inflammatory response, which was mostly made up of T lymphocytes, macrophages, and a variable amount of CD20‐positive B cells, served as the backdrop for all these alterations.^12^ It often manifests in young boys as specific neurological abnormalities such as hemiplegia, hemianesthesia, or coordination issues. Cerebellum, spinal cord, and optic chiasm involvement have also been documented.^13^

The overlap in clinical and radiological features between BCS and acute disseminated encephalomyelitis (ADEM) in this case made the diagnostic challenge even more difficult.^14^ The higher frequency of convulsions, vertigo, bilateral optic neuritis, meningismus, fever, nausea, aphasia, dysphagia, confusion, and altered levels of consciousness in ADEM can clinically distinguish it from MS despite the fact that both conditions share acute‐onset neurological symptoms and demyelinating lesions on MRI.^15^ The clinical course of BCS is variable and can be categorized into several types, including a single and self‐limited event, relapsing–remitting, and primary progressive. Historically, reports suggested a primary progressive course with a grim prognosis, often resulting in death within weeks to months. However, more recent reports have demonstrated extended survival, spontaneous remission, and even asymptomatic cases.^16^

The case presented here sheds light on the complex diagnostic challenges often encountered in the evaluation of rare neurological conditions, with a particular focus on BCS. It underscores the critical role of accurate differentiation in guiding treatment strategies and ultimately improving patient outcomes. Our patient's case highlights the intricate nature of diagnosing BCS. One of the distinguishing features of BCS is its unique concentric ring pattern on neuroimaging, which sets it apart from more common forms of MS and other demyelinating disorders.^17^ The hallmark radiological feature of BCS is the presence of alternating layers of demyelinated and preserved myelinated tissue, creating a target‐like appearance on magnetic resonance imaging (MRI) scans.^18^ This pattern of concentric rings makes me think it might be BCS, and I need more tests to tell it apart from other demyelinating diseases like ADEM. In contrast, BCS typically presents with the characteristic concentric ring pattern on MRI, while ADEM tends to exhibit more diffuse and asymmetrical lesions.^16^ In our case, the well‐defined lesions with concentric rings observed in the bilateral cerebral hemispheres prompted consideration of both BCS and ADEM.^17^

In our case, treatment with intravenous methylprednisolone, which is a common method for immune‐mediated demyelinating disorders,^19^ did not lead to the expected improvements in motor function and speech. This lack of response underscored the necessity of accurate diagnosis, as different demyelinating disorders may exhibit varied responses to similar therapeutic approaches.^20^ Although most patients have been effectively treated with immunosuppressive medications, high doses of steroids may not be able to alter the rapidly progressing clinical course of BCS. Other treatment options include plasma exchange and immunosuppressive medication, followed by autologous stem cell transplantation.^21^

This case serves as a poignant reminder of the diagnostic intricacies associated with rare neurological conditions, particularly BCS. The distinct radiological pattern of concentric rings seen on MRI imaging sets BCS apart from other demyelinating disorders, emphasizing the need for meticulous differentiation. Accurate diagnosis is paramount for tailoring appropriate treatment strategies, managing patient expectations, and estimating prognosis. Given the rarity of BCS, evidence‐based guidelines for its management are scarce, often leading to treatment strategies extrapolated from the broader literature on MS. This case also underscores the importance of interdisciplinary collaboration in neurology, emphasizing the need for further research to deepen our understanding of rare neurological disorders.

## 4 CONCLUSION

There are both common and uncommon forms of BCS. To identify the nature and potential type of MS, it is imperative that patients who arrive with symptoms consistent with MS receive the right workup and imaging. Although BCS does not have a specific treatment, a correct diagnosis aids in communicating the findings to the patient and outlining the typical course of the illness. By sharing this case report, more people will become aware of the rare MS variations, like BCS, and how important it is to consider them in the differential diagnosis despite their rarity and unusual symptoms. Additionally, we hope that our case report will contribute to the scant quantity of literature on this uncommon MS subtype and prompt additional studies to find more diagnosis‐specific treatments for BCS patients.

## AUTHOR CONTRIBUTIONS

**Mansi Singh:** Writing – original draft. **Abeer Almusleh:** Writing – original draft. **Geethika Mandru:** Writing – review and editing. **Snigdh Sahu:** Methodology. **Ogbonnaya Akuma:** Data curation. **Chinaza Mercy Akuma:** Supervision. **Brinda desai:** Software. **Archit Kumar Nigam:** Resources. **F. N. U. Sandhiya:** Investigation. **Manjeet Singh:** Writing – review and editing. **AADIL Mahmood KHAN:** Writing – review and editing.

## CONSENT

Written informed consent was obtained from the patient to publish this report in accordance with the journal's patient consent policy.

## Data Availability

The datasets analyzed during the current study are available from the corresponding author upon reasonable request. Additionally, comprehensive literature sources used for the literature review are cited appropriately within the manuscript.
